# Ta-Xi-San Suppresses Atopic Dermatitis Involved in Multitarget Mechanism Using Experimental and Network Pharmacology Analysis

**DOI:** 10.1155/2022/8441938

**Published:** 2022-05-18

**Authors:** Wenbing Zhi, Chun Li, Hong Zhang, Yiding Zhao, Shiyu Zong, Qiqi Liu, Jie Zhou, Chunliu Wang, Tingting Sun, Yang Liu, Ye Li

**Affiliations:** ^1^Shaanxi Academy of Traditional Chinese Medicine (Shaanxi Traditional Chinese Medicine Hospital), Xi'an 710003, China; ^2^Pharmacy College, Shaanxi University of Chinese Medicine, Xianyang, Shaanxi, China

## Abstract

Atopic dermatitis (AD) is a relapsing and chronic skin inflammation with a common incidence worldwide. Ta-Xi-San (TXS) is a Chinese herbal formula usually used for atopic dermatitis in clinic; however, its active compounds and mechanisms of action are still unclear. Our study was designed to reveal the pharmacological activities, the active compounds, and the pharmacological mechanisms of TXS for atopic dermatitis. Mice were induced by 2,4-dinitrocluorobenzene (DNCB) to build atopic dermatitis model. The pathological evaluation, enzyme-linked immunosorbent assay (ELISA), and hematoxylin and eosin (H&E) assay were performed. The UPLC-Q-Exactive-MS^E^ and network pharmacology analysis were performed to explore active ingredients and therapeutic mechanisms of TXS. TXS treatment decreased levels of immunoglobulin E (IgE), interleukin-4 (IL-4), and tumor necrosis factor-*α* (TNF-*α*) in serum induced by DNCB. TXS reduced scratching behavior and alleviated inflammatory pathology of skin and ear. Meanwhile, TXS decreased the spleen index and increased spleen index. The UPLC-Q-Exactive-MS^E^ results showed that 65 compounds of TXS were detected and 337 targets were fished. We collected 1371 AD disease targets, and the compound-target gene network reveled that the top 3 active ingredients were (−)-epigallocatechin gallate, apigenin, and esculetin, and the core target genes were PTGS2, PTGS1, and HSP90AA1. The KEGG pathway and GO analysis showed that TXS remedied atopic dermatitis via PI3K-Akt signaling pathway, mitogen-activated protein kinase (MAPK) signaling pathway, and Toll-like receptor (TLR) signaling pathway with the regulation of inflammatory response and transcription. Further, we found that the targets of PTGS2 and HSP90AA1 were both elevated in ears and skin of AD model mouse; however, TXS decreased the elevated expressions of PTGS2 and HSP90AA1. Our study revealed that TXS ameliorated AD based on (−)-epigallocatechin gallate, apigenin, and esculetin via targeting PTGS2 and HSP90AA1.

## 1. Introduction

Atopic dermatitis (AD) is a relapsing, intensely pruritic inflammatory disordering of the skin [1]. It is one of the most common health problems and affects 2.1%–4.9% of human population worldwide [2]. Meanwhile, the morbidity of atopic dermatitis is high in both developing countries and developed countries [3, 4]. Atopic dermatitis is characterized by rash, erythema, edema, hemorrhage, lichenification, and severe itching, and it is always accompanied by destruction in skin barriers [5]. The pathogenesis of AD is closely related to the imbalance of T helper 2 (Th2) and T helper 1 (Th1) factors [6]. Th2-based allergic inflammation plays a dominant role in the early stages of an acute outbreak of AD, which leads to the raised levels of IL-4, IL-13, and IgE [7]. However, Th1-dominant allergic inflammation is predominated in the chronic phase of AD and mainly releases IL-2, TNF-*α*, and IFN-*γ* [8, 9]. Moreover, multiple inflammatory cells are found in the epidermis and dermis of AD patients including mast cells, monocytes/macrophages, eosinophils, and T lymphocytes [10, 11].

Ta-Xi-San (TXS) is a Chinese herbal formula, consisting of six herbs: *Sophora flavescens* Aiton (*Kushen* in Chinese, KS)*, Phellodendron amurense* Rupr. (Huangbai in Chinese, HB)*, Sanguisorba* officinalis L. Bunge (*Diyu* in Chinese, DY)*, Portulaca oleracea* L. (Machixian in Chinese, MCX), *Atractylodes lancea* (Thunb.) DC. (Cangzhu in Chinese, CZ), and Alumen (Baifan in Chinese, BF), which has widely used in the Shaanxi Traditional Chinese Medicine Hospital to treat skin swelling, itching, papules, and other dermatitis symptoms for nearly 15 years. The traditional uses of TXS consist of reducing heat and expelling toxins, expelling pus and dispersing swelling, and cooling the blood and hemostasis, all of which are associated with atopic dermatitis [12–15]. In the TXS prescription, the herb of *Sanguisorba* offcinalis L. has the ability to promote wound healing, relieve pains, and reduce inflammation reactions and tissue edema [16]. The herb *Phellodendron amurense* protects human keratinocytes from PM2.5-induced inflammation and contains the bioactive compounds for atopic dermatitis management [14, 17]. The herb *Phellodendron amurense* can reduce the skin swelling and ear tissue weight of the AD mouse induced by 2,4-dinitrochlorobenzene [18]. In addition, herb of *Sophora flavescens* presents effects of anti-inflammation and antioxidant [19, 20]. Moreover, multiple active constituents in these herbs are also exhibiting anti-inflammatory and antiallergic biological activities. Oxymatrine from *Sophora flavescens* was used for AD through increasing the IL-12 and IFN-*γ* mRNA levels and reducing the ICAM-1, MDC, and SOCS1 mRNA levels [21]. Gallic acid mitigated LPS-induced inflammatory response via suppressing NF-*κ*B signaling pathway [22]. Atractylenolide I strongly inhibited 5-lipoxygenase to improve AD-like symptoms and decreased TNF-*α*, IL-6, and IL-1*β* production in lipopolysaccharide-induced acute lung jury [23, 24]. Berberine, as an index component of the *Phellodendron amurense*, suppressed the release of IL-6, CXCL8, and chemotactic factors in the eosinophils-dermal fibroblasts coculture [25]. However, the active constituents, molecular targets, and inherent pathways of TXS are rarely reported for AD treatment. Therefore, our study was designed for illustrating pharmacological effects and potential mechanisms.

Network pharmacology has made a significant contribution to systematically reveal the function and behavior between herbal formulas [26]. This research method systematically revealed effects and the potential mechanisms of multicomponent formula, through analyzing chemical component-target interaction networks [27]. Its dynamic and systematic characteristics are coincided with the theory of traditional Chinese medicine (TCM), which was suited for exploring the compound system of TCM with multiple components and multiple targets. The 63 constituents of the XIAOPI formula which prevents the breast cancer development were successfully found and validated based on network pharmacology [28]. Thus, we used AD mice model induced by DNCB to analyze efficacy of TXS and applied UPLC-Q-Exactive-Ms^E^ and network pharmacology study to illuminate potential mechanism of TXS.

## 2. Materials and Methods

### 2.1. Materials and Reagents

TXS was obtained from Shaanxi Academy of Traditional Chinese Medicine. Methanol and formic acid (LC-MS-grade) were purchased from Thermo Fisher Scientific Co., Ltd. (Waltham, MA, USA). 2,4-Dinitrofluorobenzene (DNCB) was purchased from Macklin Biochemical Technology Co., Ltd. Hydrocortisone Butyrate Cream was obtained from Hunan WZT Pharmaceutical Co., Ltd. (Xiangtan, China). The rat IL-4, TNF-*α*, and IgE ELISA kits were obtained from Nanjing Keygen Biotech (Nanjing, China). PTGS2 and HSP90AA1 ELISA kits were purchased from R&D (Minneapolis, MN, USA).

### 2.2. TXS Preparation

TXS (160 g, Shaanxi Academy of Traditional Chinese Medicine) was soaked with 1000 mL in water for 30 min, decocted for 5 min again after boiled, and then filtrated. The decoction filtrated was concentrated to 160 mL (1 g crude drug/mL). The solution was filtered using 0.22 mm membranes. The filtrate was used and stored at 4°C before its use for animal assays.

### 2.3. Building Atopic Dermatitis Mice Model and Treatment

BALB/c mice (male, 18–20 g) were purchased from Xi'an Jiao Tong University (Xian, China). All the mice were fed under the standard experimental conditions (−25 ± 2°C, humidity 60 ± 5%, and 12/12 h day/night cycle). The AD mice model was induced by DNCB (dissolved in acetone/olive oil (3 : 1)), which was applied to dorsal skin and ear. Mice were segmented into 6 groups (*n* = 6 per group): (1) normal group, (2) matrix group, (3) DNCB model group, (4) DNCB + matrix + 0.65 mg crude drug/mL TXS, (5) DNCB + matrix + 1.30 mg crude drug/mL TXS, and (6) Hydrocortisone Butyrate Cream (Hyd B). Firstly, the mice were shaved with an aesthetic state (ethyl carbamate) using an electric shaver. Then, 100 *μ*L 0.5% DNCB or acetone/olive oil (3 : 1) was applied to the shaved dorsal skin for 2 days, and there was no treatment in the 3rd∼6th days . 70 *μ*L 0.5% DNCB on dorsal skin and 20 *μ*L 0.5% DNCB on ear every 2 days were applied from the 7th day. The AD model was finished on the 28th day for a total of 10 times (on days 1, 2, 7, 10, 13, 16, 19, 22, 25, and 28). DNCB was applied on the same site *r*. TXS was applied from the 7th day, 500 *μ*L on dorsal skin and 200 *μ*L on ears, twice a day until the 28th day. Hyd B was also applied from the 7th day, 300 mg on dorsal skin and 70 mg on ears, twice a day until the 28th day. The flowchart of the experimental program we studied is shown in Figure 1. Our animal study followed the guidelines (Care and Use of Laboratory in Xi'an Jiao Tong University Health Science Center, license approval no. SCXK (Shan) 2017-003).

### 2.4. Evaluation of Skin Lesion and Measurement of Ear Weight

The relative severity of AD was evaluated weekly via scoring the lesions of the dermal tissues with the scoring procedure [29]: (1) erythema and hemorrhage, (2) erosion (excoriation), (3) edema, and (4) scaling (dryness). In each score, 0 was defined as exhibiting no symptoms, 1 as mild symptoms, 2 as moderate symptoms, and 3 as severe symptoms. Only one researcher participated in scoring the apparent AD symptoms throughout the experiment to minimize technique variations. The ears of each mouse were harvested and weighted.

### 2.5. The Thymus Index and Spleen Index Measurement

The spleen and thymus of mice in each group were removed integrally. The thymus index and spleen index were defined as the organ/body ratio (organ mass (mg)/corresponding animal mass (g)). The organ and the body weight were calculated using an electronic balance.

### 2.6. Histological Analysis

The dorsal skin and ear samples were taken 24 h after final herbal administration and then fixed in 4% paraformaldehyde buffer, followed by embedding of the tissues in paraffin wax. The tissue sections were 2 *μ*m thick, and then they were stained with H&E.

### 2.7. Cytokines Quantitation

Total IgE in serum was analyzed using an ELISA Quantitation Kit according to the manufacturer's protocol. The serum concentrations of the cytokines, including TNF-*α* and IL-4, were also quantified using a mouse cytokine enzyme immunoassay kit, respectively.

### 2.8. UPLC-Q-Exactive-MS^E^ Analysis

The TXS aqueous extract was analyzed with a 150 mm × 2.1 mm Accucore AQ C18 column (2.6 *μ*m). The mass spectrometer used in the UPLC-Q-Exactive-MS^E^ analysis was a quadrupole-electrostatic field orbital with an ESI mode and data treating used Mass Lynx 4.1 software. Column temperature was 30°C. The mobile phase consisted of 2 solvents: (A) 0.1% formic acid aqueous solution and (B) methyl alcohol (for a gradient elution program: 0–10 min, 95% solvent A; 20–30 min, 75% solvent A; 35 min, 30% solvent A; 45–60 min, 5% solvent A; 60–65 min, 95% solvent A). The flow rate was kept at 0.3 mL/min. The injection volume was set as 1 *μ*L. The ion source of thermoelectric spray (HESI) MS was performed to collect data in full switch ion mode. Other parameters were as follows: capillary temperature: 300°C, auxiliary gas heater: 300°C, sheath gas flow rate: 30 L/min, spray voltage: 3.50 kV, full MS resolution: 7000, ddms2 resolution: 175000, and scan range: 100 to 1 200 Da. S-lens RF level was set as 55 V.

### 2.9. Network Pharmacology Study

#### 2.9.1. Fishing Targets

In this work, we search the targets of UPLC-Q-Exactive-MS^E^ analysis ingredients of TXS based on Traditional Chinese Medicine System Pharmacology Database and Analysis Platform (TCMSP, https://lsp.nwu.edu.cn/tcmsp.php) and the Comparative Toxicogenomics Database (CTD, https://ctd.mdibl.org/) based on UPLC-Q-Exactive-MS^E^ analysis. The UniProt (https://www.uniprot.org/) database was used for drug target revision to match the official name. The Online Mendelian Inheritance in Man (OMIM, https://www.omim.org/), Comparative Toxicogenomics Database (CTD, https://ctd.mdibl.org/) and GeneCards-Human Genes (GeneGards: https://www.genecards.org/) database were used to collect the AD-related disease genes.

#### 2.9.2. Network Construction

For better dissecting the latent active ingredients and key targets of TXS, we established the herb-ingredient-target-pathway network using Cytoscape 3.7.1 software. Then, the quantitative “degree” was analyzed by plugin network analyzer. According to the descending order of “degree,” we selected the vital ingredients and targets of TXS against AD.

#### 2.9.3. Functional Enrichment Assay

The Gene Ontology (GO) enrichment and the Kyoto Encyclopedia of Genes and Genomes (KEGG) pathway (https://www.genome.jp/kegg/pathway.html) assay was performed based on the clusterProfiler software package on *R* platform and analyzed using visualization. Afterwards, the GO interactive network and the bubble diagram of KEGG pathway were structured using the top GO packet of *R* platform. *P* < 0.05 was calculated meaningfully in these two enrichment analyses.

### 2.10. Targets Verification

To identify the targets of TXS on AD treatment, we performed the ELISA assay. The protein expressions of PTGS2 and HSP90AA1 were quantitated. In brief, the ears and skin were fully ground with RIPA buffer adding 0.1 M PMSF and phosphatase inhibitors. Then, the supernatant was collected via centrifugation at 10000 rpm for 15 min at 4°C. The PTGS2 and HSP90AA1 expressions in supernatant were quantified using a mouse ELISA kit (R&D Systems, Minneapolis, MN, USA).

### 2.11. Statistical Analysis

Our data are shown as the mean ± standard deviation (SD). Statistical comparison among groups was analyzed with GraphPad Prism 5.01 (California, USA). ANOVA was firstly used followed by Student's *t*-test. *P* < 0.05 indicated significant difference between groups.

## 3. Result

### 3.1. TXS Alleviates the Lesions in Ear and Back

The skin inflammation of the back and ear of mice in each group was observed by visual method (Figure 2(a)). The skin of the ear and back of normal mice was smooth and healthy. Compared with the normal mice, the ear of mice in DNCB group was obviously swollen, rough, desquamate, and auricle with scab. Meanwhile, the back skin of mice in model group was thickened, rough, erythema, desquamate, and scab, which showed a typical dermatitis feature. However, TXS dramatically decreased the excoriation, striking hemorrhage, and erosion and suppressed the scratching behavior compared to the DNCB-induced mice. In addition, in HYB treatment group, the inflammatory response was lighter, the damage and scratches just existed in edge of the ear, the back skin was thinner, and the vascular lines were clear.

At the same time, the lesion of back skin was scored according to the “inflammatory score standard.” Compared with the normal mice, the back inflammatory score of mice in DNCB group was significantly enhanced, and TXS (1.3 mg crude drug/mL) significantly reduced the inflammatory score (Figure 2(b)). There was a significant increase in ear weight of mice in DNCB group due to swelling of the ear compared with the mice in the normal group (Figure 2(c)). TXS and HBY administration decreased the ear weight and back of mice, respectively. In conclusion, both TXS and HYB promoted inflammation subsidence and skin healing of mice.

### 3.2. TXS Improved the Thymus Index and Spleen Index

As Figures 3(a) and 3(b) show, compared with the normal group, the thymus index of mice in DNCB group was memorably reduced; TXS administration could improve the thymus index of mice. The spleen index of DNCB-stimulated mice was significantly higher than that in the normal mice. High-dose TXS administration effectively reduced the spleen index.

### 3.3. Histological Analysis Results

Hematoxylin study was used to recognize whether TXS regulates pathological symptoms of AD-like skin lesions and ear injury in DNFB-induced AD mouse model. In model group, skin tissues of mice showed typical inflammatory pathological changes including parakeratosis, thickening of the spinous layer, telangiectasia, and infiltration of inflammatory cells in the dermis (Figure 4(a)). In mice in TXS and HYB treatment group, there was no parakeratosis in skin tissue, and the spinous layer was thickened; however, a trifling infiltration of inflammatory cell was still in the dermis (Figure 4(a)). Meanwhile, ear histological analysis showed that TXS decreased the epidermal thickening and inflammatory cells accumulation in the lesions (Figure 4(b)).

### 3.4. TXS Regulated the Level of Cytokines

Elevated levels of inflammatory cytokines and inflammatory cell infiltration are a typical characteristic in AD [30]. Thus, we estimated the cytokines level in the serum of DNFB-sensitized mice. Subsequently, we observed that the TXS has an effect on the release of inflammatory factors. The levels of IL-4, TNF-*α*, and IgE in serum were significantly increased in the model group's mice induced by DNFB compared to the normal group. However, production of IL-4, TNF-*α*, and IgE was inhibited by TXS and Hyd B treatment (Figures 5(a)–5(c)).

### 3.5. The Ingredients Analysis of TXS Extracts

The herb components of TXS extracts were detected via aligning each detectable compound mass data for each detectable compound with structure and confirmed by MS^E^ substructure data. The Base Peak Chromatogram (BPC) of TXS extracts in positive ion mode and negative ion mode is shown in Figures 6(a) and 6(b). TXS mainly contained alkaloids and flavonoid glycosides, and these ingredients presented a better MS response in positive than in the positive ion mode. In this research, 65 compounds extracted in TXS were identified through comparing and analyzing the primary and secondary mass spectrometry information, combining with databases (Metlin, Massbank, and Human Metabolome Database) and combining with retention behavior, database, and related literature reports. The 65 compounds were confirmed as the principal compounds for the following assay and are detailedly displayed in Table 1.

### 3.6. Potential Target Genes and Network Analysis

The 337 targets were collected form the 65 compounds in TXS based on UPLC-Q-Exactive-MS^E^ analysis after eliminating the duplicate targets. Simultaneously, 1371 AD-related targets were collected via searching CTD, GeneCards, and OMIM databases, and 1241 targets were decontaminated after removing duplicates. Then the compound targets and disease-related targets were merged, and we got the compound-target gene network.

The ingredient-target gene network is presented in Figure 7. This network consisted of 190 nodes (1 TXS formula node, 52 compounds, and 137 target genes) and 522 edges. Compounds in the network were classified as catechin class, flavonoids, coumarin, isoflavone, and alkaloids. Particularly, as shown in Tables 2 and 3, the top five ingredients of TXS which have maximum degrees are (−)-epigallocatechin gallate, apigenin, esculetin, wogonin, and epicatechin. Additionally, 27 genes (ADH1C, ADRA1B, IL-4, RELA, TP53, TOP2A, TNF, RXRA, PTGS2, PTGS1, PRKACA, PPARG, PIK3CG, NOS3, NOS2, NFKBIA, MAOA, JUN, HSP90AA1, ESR1, CDKN1A, CCND1, CASP3, BCL2, AR, AKT1, and ADRB2) were recognized due to their interactions with more than five ingredients. The ingredient-target gene network contributed to understanding the possible effects of TXS.

### 3.7. The Results of KEGG and GO Analysis

KEGG pathway enrichment showed that 199 pathways were harvested and the remarkable 30 related pathways are presented in Figure 8(a). Pathways in PI3K-Akt signaling pathway, MAPK signaling pathway, and TNF signaling pathway may be the latent mechanism to exert effects of TXS against AD. Subsequently, the results of GO evaluation of the top 10 enriched results are shown in Figure 8(b). The enriched biological process ontologies were dominated by positive regulation of transcription from RNA polymerase II promoter, negative regulation of apoptotic process, response to drug, inflammatory response, and positive regulation of transcription. The molecular function of targets was mainly enriched in ontologies including protein binding, identical protein binding, protein homodimerization activity, and enzyme binding. Meanwhile, cell component result showed that cytoplasm is the largest constitution.

### 3.8. TXS Regulated the PTGS2 and HSP90AA1 Expressions in Mouse Model

PTGS2 and HSP90AA1 are major regulatory targets for inflammatory response in AD and are core targets screened via network pharmacology. Thus, we investigate the regulatory effect of TXS on activation of PTGS2 and HSP90AA1. In our study, we found that the protein expressions of PTGS2 and HSP90AA1 in ears and skin of model mice were significantly enhanced compared to the normal mice; however, TXS decreased the elevated expressions of PTGS2 and HSP90AA1 (Figures 9(a)–9(d)). Our results revealed that TSX might be a useful drug for AD therapy via regulating PTGS2 and HSP90AA1 expressions.

## 4. Discussion

The DNCB-induced skin lesion in mice is a classical animal model for AD research [31]. Thus, we established DNCB-induced mouse model to assess the effects of TXS on AD. IL-4 and TNF-*α* are risk factors for developing atopic dermatitis [32]. Previous studies showed that cytokines including IL-4, TNF-*α*, and IL-1*β*-were enhanced in serum of AD patients [33]. Higher level of IFN-*γ* and IL-6 was detected in skin lesions of AD patients [34]. In our study, the levels of IL-4, TNF-*α*, INF-*γ*, and IgE in serum were reduced; meanwhile, the inflammation of back skin, the skin inflammation score, and the ear swelling of mice were alleviated after taking the TXS. Hence, TXS might be effective to balance atopic and inflammatory disorders in the progress of atopic dermatitis.

In addition, to explore the effects of TXS on skin and ear inflammation, we performed H&E assay and examined thymus index and spleen index. The mice induced by DNFB showed typical AD features, such as epidermal hyperplasia and massive inflammatory cells infiltration, which were coincided with the typical symptoms of AD. TXS treatment effectively improved the skin and ear status. The thymus is a major immune organ, the index of which is an important index for assessing immunity [35]. Meanwhile, as another lymphatic organ of the human body, the spleen palys a core role in immune system and is used for assessing immunomodulatory effects of drugs [36]. TXS treatment lowered the spleen index and enhanced the thymus index. Therefore, TXS regulated pathological changes in the development of AD.

UPLC-Q-Exactive-MS^E^ as a rapid, efficient, and sensitive method is always used for analyzing extracts and bioactive ingredients from medicine and herbs [37, 38]. Therefore, we applied UPLC-Q-Exactive-Ms^E^ to analyze the information on compounds in herbal medicines of TXS. 65 components in TXS were identified, including alkaloids, phenols, flavonoids, and acids. Among them, various ingredients showed anti-inflammatory activity. Matrine, a quinolizidine alkaloid extracted from *Sophora flavescens*, has the capacity to effectively suppress experimental autoimmune encephalomyelitis and optic neuritis [39, 40]. Oxyberberine prevented lipopolysaccharide-induced acute lung injury and improved colitis [41, 42]. Epicatechin from *garden burnet*, epiberberine from *golden cypress*, and atractylenolide I from *Rhizoma atractylodis* showed anti-inflammatory activity [43–45]. Thus, we predict that TXS has an anti-inflammatory material basis.

The network pharmacology study as a major tool systematically revealed the effects and mechanism of multicomponent and multitarget system, such as traditional Chinese medicine [46, 47]. Here, we researched the pharmacological mechanisms of TXS against atopic dermatitis through using the network analysis method. The ingredient-target gene network pharmacological analysis of TXS identified 52 ingredients and 137 target genes connected with AD. That means that one chemical component acted with an average of 9.03 targets, while one target was bound with an average of 3.43 compounds. The compound-target gene network of TXS revealed that (−)-epigallocatechin gallate (degree = 61, CC = 0.4797, BC = 0.3317), apigenin (degree = 41, CC = 0.4355, BC = 0.1750), and esculetin (degree = 34, CC = 0.4219, BC = 0.1296) were the major pharmacodynamic compositions of TXS according to the degree. Epigallocatechin gallate is a single ingredient from TCM and shows effective functions against AD due to the antioxidant and immunomodulatory effects [48]. Apigenin inhibits inflammatory cytokines (IL6, TNF-*α*, IL-5, and IL-13) production to decrease allergic responses in RBL-2H3 cells and repairs the physical barrier of the skin in HaCaT cell model [49]. Esculetin attenuates atopic skin inflammation by inhibiting IFN-*γ*, IL-13, IL-31, and IL-17 release via regulating nuclear factor-*κ*B pathway [50]. Furthermore, in this network, the first 3 targets of degree values were PTGS2 (degree = 41, CC = 0.4846, BC = 0.1297), PTGS1 (degree = 27, CC = 0.3873, BC = 0.0358), and HSP90AA1 (degree = 21, CC = 0.3691, BC = 0.0224). Meanwhile, the three targets with higher BC and CC were recognized as critical targets of TXS for AD treatment. Thus, our results indicated that TXS as the complex system of herbal compounds displayed multipharmacological and superimposed effects.

Based on the enrichment results of KEGG, we determined that the effects of TSX against AD may be due to pathways like PI3K-Akt signaling pathway, MAPK signaling pathway, Th17 cell differentiation, and TLR signaling pathway. The mitogen-activated protein kinase (MAPK) pathway is responsible for inflammatory and immune response and is widely expressed in multiple tissues [51]. Previous study showed that *Solanum nigrum* Linne possessed anti-inflammatory effects in vitro through regulating MAPK/NF-*κ*B pathway in HaCaT cell model [52]. It has been reported that inhibiting TLR signaling pathway was a critical approach for chronic allergic skin inflammation treatment [53]. *Artemisia argyi* Folium extract ameliorates DNCB-induced skin lesions in BALB/c mice via inhibiting PI3K/Akt pathway [54]. In this study, target genes enrichment was mainly associated with the biological processes including positive regulation of transcription from RNA polymerase II promoter, negative regulation of apoptotic process, inflammatory response, and positive regulation of transcription. Further, enriched MF ontologies were dominated through protein binding, enzyme binding, identical protein binding, and protein homodimerization activity. In addition, CC analysis displayed that cytoplasm was the largest constitution. Further, we found that TXS downregulated the expressions of PTGS2 and HSP90AA1. More importantly, the center target HSP90AA1 selected by the compound-target gene network was involved in the PI3K-Akt signaling pathway and PTGS2 was the major target for anti-inflammation.

## 5. Conclusions

In conclusion, our results revealed that TXS attenuated IL-4, IgE, and TNF-ɑ levels in serum, increased thymus index, and decreased spleen index. TXS ameliorated behavioral changes and alleviated pathological changes of skin and ear in mice with the DNCB-induced atopic dermatitis. Additionally, TXS was mainly consisted of 65 chemical components. Among them, 52 components were closely associated with the effect of TXS against AD. TXS downregulated PTGS2 and HSP90AA1, which were associated with the PI3K-Akt signaling pathway. Our results revealed the effects, components, and pharmacological mechanism of TXS for AD, which provided scientific basis for clinical application.

## Figures and Tables

**Figure 1:** The schematic diagram of modeling method and treatment.

**Figure 2:** The morphological observation and assessment. (a) The morphological changes of skin and ears. (b) Inflammation score of skin. (c) The ear weight value. Values are expressed as mean ± SD (*n* = 6). ^*∗*^*P* < 0.05 and ^*∗∗*^*P* < 0.01 compared with the normal group; ^^^*P* < 0.05 and ^^^^*P* < 0.01 compared with the matrix group; ^#^*P* < 0.05 and ^##^*P* < 0.01 compared with the DNFB model group.

**Figure 3:** TXS regulates the thymus index and the spleen index. (a) The assessment of the thymus index. (b) The assessment of the spleen index. Values are expressed as mean ± SD (*n* = 6). ^*∗*^*P* < 0.05 and ^*∗∗*^*P* < 0.01 compared with the normal group; ^^^*P* < 0.05 and ^^^^*P* < 0.01 compared with the matrix group; ^#^*P* < 0.05 and ^##^*P* < 0.01 compared with the DNFB model group.

**Figure 4:** TXS inhibits inflammation of skin and ears. ((a) and (b)) Hematoxylin and eosin- (H&E-) stained sections of skin tissues. Magnification x4.

**Figure 5:** TXS decreases cytokines in serum. (a) The level of IL-4 in serum was determined by ELISA. (b) The level of TNF-*α* in serum was determined by ELISA. (c) The IgE production in serum was calculated by ELISA. Values are expressed as mean ± SD (*n* = 6). ^*∗*^*P* < 0.05 and ^*∗∗*^*P* < 0.01 compared with the normal group; ^^^*P* < 0.05 and ^^^^*P* < 0.01 compared with the matrix group; ^#^*P* < 0.05 and ^##^*P* < 0.01 compared with the DNFB model group.

**Figure 6:** The detection of chemical components in TXS. (a) UPLC-Q-Exactive-MS^E^ total ion current chromatogram of TXS under positive ion mode. (b) UPLC-Q-Exactive-MS^E^ total ion current chromatogram of TXS under negative ion mode.

**Figure 7:** The component-targets network of TXS against AD.

**Figure 8:** The mechanism exploration of TXS against AD. (a) KEGG pathway enrichment analysis of the TXS predicted targets. Bubble diagram of the top 30 KEGG pathways. (b) The top 5 GO analysis terms for CC, BP, and CF with the most significant *P* values of targets in AD.

**Figure 9:** TXS alleviated AD via targeting PTGS2 and HSP90AA1. (a) The PTGS2 expression in ears was determined by ELISA. (b) The PTGS2 expression in skin was determined by ELISA. (c) HSP90AA1 in ears was calculated by ELISA. (d) HSP90AA1 in skin was calculated by ELISA. Values are expressed as mean ± SD (*n* = 6). ^*∗*^*P* < 0.05 and ^*∗∗*^*P* < 0.01 compared with the normal group; ^^^*P* < 0.05 and ^^^^*P* < 0.01 compared with the matrix group; ^#^*P* < 0.05 and ^##^*P* < 0.01 compared with the DNFB model group.

**Table 1:** The chemical composition analysis of TXS decoction by UPLC-Q-Exactive-MS^E^

No.	Compound	Area	RT (means)	Formula	Measure m/z	Fragmentation	Delta m/z	Adducts	±	Sources
1	Matrine	1980000000	4.42	C_15_H_24_N_2_O	249.2	70.065, 84.0868, 152.1433	−2.46	H		KS
2	Oxysophocarpine	1200000000	6.22	C_15_H_22_N_2_O_2_	263.18	—	−1.68	H	+	KS
3	7-Demethylsuberosin	139000	36.68	C_14_H_14_O_3_	253.08	55.0545, 69.0699, 83.0854	−4.13	Na	+	KS
4	Kurarinone	948000	38.38	C_26_H_30_O_6_	461.19	—	−1.54	Na	+	KS
5	Kushenol F	939000	39.72	C_25_H_28_O_6_	423.18	—	0.13	H	−	KS
6	Trifolirhizin	118000000	36.85	C_22_H_22_O_10_	469.11	149.0228, 193.0491, 237.0754	−1.2	Na	+	KS
7	Xanthohumol	836000	37.48	C_21_H_22_O_5_	353.14	112.9856, 129.9757, 248.9604	−0.13	Na	−	KS
8	Isoxanthohumol	3600000	37.49	C_21_H_22_O_5_	377.14	92.5511, 192.9041, 203.1646	−1.33	Na	+	KS
9	Oxymatrine	2.87*E* + 09	7.38	C_15_H_24_N_2_O_2_	265.19	136.112, 205.1333, 247.1802	−2.45	H	+	KS
10	Methylparaben	354000000	1.53	C_12_H_16_N_2_O	205.13	58.0653, 91.0539, 146.0602	−1.84	H	+	KS
11	Formononetin	5670000	37.05	C_16_H_12_O_4_	291.06	\	−1.7	H	+	KS
12	Sophocarpine	370000000	7.42	C_15_H_22_N_2_O	247.18	98.0599, 150.1276, 148.1118	−1.58	H	+	KS
13	Neochlorogenic acid	5300000	18.35	C_16_H_18_O_9_	355.1	92.5453, 120.9673, 142.9385	−1.82	H	+	HB
14	Palmatine	80100000	34.85	C_21_H_22_NO_4_	352.15	127.1117, 327.2526, 377.2648	−1.91	H	+	HB
15	Oxyberberine	25000000	27.16	C_20_H_17_NO_5_	352.12	62.1674, 79.1569, 138.1779	−1.73	H	+	HB
16	Tetrahydropalmatine	60200000	22.48	C_21_H_25_NO_4_	356.19	149.012, 167.0225, 315.1926	−1.35	H	+	HB
17	Rutaevin	3940000	16.31	C_26_H_30_O_9_	504.22	116.9857, 134.9963, 164.9843	−1.33	NH4	+	HB
18	Epiberberine	6320000000	34.6	C_20_H_18_NO_4_	337.12	149.012, 167.0225, 307.1769	−2.58	H	+	HB
19	Phellodendrine	1210000000	44.75	C_20_H_24_NO_4_	343.17	66.6729, 84.9595, 126.2253	−2.31	H	+	HB
20	Berberine	6320000000	39.32	C_20_H_18_NO_4_	337.12	79.9573, 96.96, 309.1704	−2.58	H	+	HB
21	Coniferin	5470000	16.79	C_16_H_22_O_8_	365.12	116.9857, 149.012, 164.9843	−1.49	H	+	HB
22	Vanillin	9890000	18.37	C_8_H_8_O_3_	153.05	105.0031, 116.9857, 149.0119	−0.56	H	+	HB
23	Paeonol	35700000	38.34	C_9_H_10_O_3_	167.07	56.965, 116.9857, 167.0025	−0.84	H	+	HB
24	Isovanillin	9890000	18.37	C_8_H_8_O_3_	153.05	—	−0.56	H	+	HB
25	Berberrubine	17900000	33.67	C_19_H_15_NO_4_	322.11	79.9055, 242.4609, 269.4887	−1.39	H	+	HB
26	Ethyl caffeate	1990000	22.86	C_11_H_12_O_4_	209.08	72.0835, 80.518, 105.3846	1.68	H	+	HB
27	Limonin	101000000	35.78	C_26_H_30_O_8_	493.18	88.3646, 250.7163, 350.8599	−1.86	H	+	HB/CZ
28	Ferulic acid	387000	40.09	C_10_H_10_O_4_	195.07	65.0387, 95.049, 121.0282	−0.41	H	+	HB
29	Esculetin	1570000	16.43	C_9_H_6_O_4_	177.02	58.9718, 90.998, 94.993	−0.24	H	−	HB
30	L-Adenosine	39200000	2.22	C_10_H_13_N_5_O_4_	268.1	94.0397, 119.0351, 136.0617	−1.8	H	+	HB
31	Tetrahydroberberine THB	1930000	21.77	C_20_H_21_O_4_N	340.15	64.0373, 142.9384	−1.17	H	+	HB
32	Berbamine	295000	36	C_37_H_40_N_2_O_6_	609.29	—	−2.32	H	+	HB
33	Jatrorrhizine	347000	42.29	C_20_H_20_NO_4_	339.15	64.0373, 142.9384	0.55	H	+	HB
34	Gallic acid	139000000	2.45	C_7_H_6_O_5_	169.01	69.0345, 97.0294, 125.0249	−0.98	H	−	DY
35	Gallic acid trimethyl ether	2260000	31.94	C_10_H_12_O_5_	213.08	—	−1.1	H	+	DY
36	(−)-Epigallocatechin gallate	277000	21	C_22_H_18_O_11_	457.08	—	−1.45	H	−	DY
37	Epigallocatechin	4470000	1.53	C_15_H_14_O_7_	307.08	93.8318, 122.1348, 174.7394	4.4	H	+	DY
38	Brevifolincarboxylic acid	446000	20.04	C_13_H_8_O_8_	315.01	106.3279, 210.9946, 310.6447	−1.36	Na	+	DY
39	(−)-Epicatechin gallate	6400000	1	C_22_H_18_O_10_	441.08	79.9573, 94.9808, 96.96	−1.01	H	−	DY
40	Epicatechin	80300000	15.85	C_15_H_14_O_6_	289.07	97.0294, 109.0294, 123.0451	−0.57	H	−	DY
41	Protocatechuic acid	2660000	4.88	C_7_H_6_O_4_	153.02	—	−0.58	H	−	DY
42	Methyl gallate	2920000	8.55	C_8_H_8_O_5_	183.03	79.9573, 95.9522, 118.9419	−0.71	H	−	DY
43	Procyanidin B1	16600000	14.89	C_30_H_26_O_12_	577.14	55.9346, 72.937, 90.9476	−0.24	H	−	DY
44	Procyanidin B2	16600000	14.89	C_30_H_26_O_12_	577.14	55.9346, 72.937, 90.9476	−0.24	H	−	DY
45	Ethyl gallate	13400000	21.71	C_9_H_10_O_5_	197.05	96.9601, 128.0352, 152.895	−0.25	H	−	DY
46	Ellagic acid	1020000	34.79	C_14_H_6_O_8_	301	—	0.52	H	−	DY
47	Hyperoside	308000	40.62	C_21_H_20_O_12_	465.1	—	0.86	H	+	DY
48	Ursonic acid	26600000	37.47	C_30_H_46_O_3_	455.35	107.9667, 192.0492, 236.9945	−1.03	H	+	DY
49	Cianidanol	80300000	15.85	C_15_H_14_O_6_	289.07	97.0294, 109.0294, 123.0451	−0.57	H	−	DY
50	Atractylodin	16400000	37.6	C_13_H_10_O	183.08	91.0541， 95.0490， 119.0490	−0.89	H	+	CZ
51	Atractylenolide II	40400000	38.09	C_15_H_20_O_2_	255.14	55.0545, 69.0699, 83.0854	−1.4	Na	+	CZ
52	Atractylenolide I	2150000	37.76	C_15_H_18_O_2_	254.12	55.0545, 69.0699, 81.0197	−0.09	H	+	CZ
53	Wogonin	11500000	35.27	C_16_H_12_O_5_	285.08	—	−1.41	H	+	CZ
54	Baicalin methyl ester	4180000	36.9	C_22_H_20_O_11_	283.09	—	−1.19	Na	+	CZ
55	Atractyloside A	27400000	36.27	C_21_H_36_O_10_	471.22	64.023, 190.5318, 350.8599	−1.57	Na	+	CZ
56	Vanillic acid	488000	1.01	C_8_H_8_O_4_	169.05	59.965, 57.935, 84.9586	−1.59	H	+	CZ
57	Protocatechualdehyde	3620000	37.47	C_7_H_6_O_3_	139.04	72.9370, 97.0074, 111.0231	−0.43	H	+	CZ
58	Citric acid	327000000	0.96	C_6_H_8_O_7_	191.02	85.0295, 87.0086, 111.0087	−0.4	H	−	MCX
59	Benzoic acid	82900000	1.75	C_7_H_6_O_2_	123.04	65.0386， 77.0384， 95.0490	−1.49	H	+	MCX
60	Caffeic acid	23200000	40.11	C_9_H_8_O_4_	181.05	95.0490, 103.0540, 121.0646	−1.32	H	+	MCX
61	Apigenin	2230000	36.31	C_15_H_10_O_5_	269.05	—	0.05	H	−	MCX/KS
62	Allantoin	2830000	0.99	C_4_H_6_N_4_O_3_	159.05	57.0700， 91.0541， 115.0546	−0.96	H	+	MCX
63	Isoscopoletin	3950000	37.01	C_10_H_8_O_4_	193.05	133.052, 148.0755, 191.1195	−0.76	H	+	MCX
64	Mannitol	14000000	0.97	C_6_H_14_O_6_	205.07	56.0497，58.0653,146.0602	−2.05	H	+	MCX
65	Scopolin	24500000	18.28	C_16_H_18_O_9_	377.08	92.5511， 129.6406， 203.1646	−1.57	H	+	MCX

*Note*: KS stands for *Sophora flavescens*; HB stands for *Phellodendron amurense*; DY stands for *Sanguisorba officinalis* L.; CZ stands for *Atractylodes lancea*; MCX stands for *Portulaca oleracea.*

**Table 2:** The pharmacodynamic compounds of TXS for AD.

No.	Compound	Betweenness centrality (BC)	Closeness centrality (CC)	Degree
1	(−)-Epigallocatechin gallate	0.3317	0.4797	61
2	Apigenin	0.1750	0.4355	41
3	Esculetin	0.1296	0.4219	34
4	Wogonin	0.0668	0.4127	29
5	Epicatechin	0.0483	0.3954	19
6	Formononetin	0.0371	0.39375	18
7	Oxymatrine	0.0714	0.3889	15
8	Ellagic acid	0.0459	0.3873	14
9	Paeonol	0.0200	0.3873	14
10	Caffeic acid	0.0457	0.3857	13

**Table 3:** The pharmacodynamic targets of TXS for AD.

No.	Target	Betweenness centrality (BC)	Closeness centrality (CC)	Degree
1	PTGS2	0.12968939	0.48461538	41
2	PTGS1	0.03576985	0.38729508	27
3	HSP90AA1	0.02247622	0.36914063	21
4	ESR1	0.0193549	0.38259109	15
5	PRKACA	0.00849434	0.34615385	14
6	RXRA	0.00732045	0.32926829	14
7	NOS2	0.01528486	0.37951807	12
8	ADRB2	0.00526221	0.32363014	11
9	TNF	0.03753438	0.42376682	11
10	TOP2A	0.00637523	0.33392226	11

## Data Availability

All the data used to support the findings of this study are submitted and are available in this published article.

## Abbreviations

AD: Atopic dermatitis
TXS: Ta-Xi-San
DNCB: 2,4-Dinitrofluorobenzene
Th2: T helper 2
GO: Gene Ontology
IL: Interleukin
KEGG: Kyoto Encyclopedia of Gene and Genomics
LPS: Lipopolysaccharide
MAPK: Mitogen-activated protein kinase
NF: Nuclear factor
PPI: Protein-protein interaction
QTOF: Quadrupole-time of flight
TNF: Tumor necrosis factor
UPLC: Ultraperformance liquid chromatography
PTSG: Prostaglandin G/H synthase.
